# The Microenvironment That Regulates Vascular Wall Stem/Progenitor Cells in Vascular Injury and Repair

**DOI:** 10.1155/2022/9377965

**Published:** 2022-07-31

**Authors:** Ying Ma, Yuan Li, Yan Yang, Pengyun Li

**Affiliations:** Key Laboratory of Medical Electrophysiology of Ministry of Education and Medical Electrophysiological Key Lab of Sichuan Province, Collaborative Innovation Center for Prevention and Treatment of Cardiovascular Disease, Institute of Cardiovascular Research, Southwest Medical University, Luzhou, 646000 Sichuan, China

## Abstract

Vascular repair upon injury is a frequently encountered pathology in cardiovascular diseases, which is crucial for the maintenance of arterial homeostasis and function. Stem/progenitor cells located on vascular walls have multidirectional differentiation potential and regenerative ability. It has been demonstrated that stem/progenitor cells play an essential role in the basic medical research and disease treatment. The dynamic microenvironment around the vascular wall stem/progenitor cells (VW-S/PCs) possesses many stem cell niche-like characteristics to support and regulate cells' activities, maintaining the properties of stem cells. Under physiological conditions, vascular homeostasis is a cautiously balanced and efficient interaction between stem cells and the microenvironment. These interactions contribute to the vascular repair and remodeling upon vessel injury. However, the signaling mechanisms involved in the regulation of microenvironment on stem cells remain to be further elucidated. Understanding the functional characteristics and potential mechanisms of VW-S/PCs is of great significance for both basic and translational research. This review underscores the microenvironment-derived signals that regulate VW-S/PCs and aims at providing new targets for the treatment of related cardiovascular diseases.

## 1. Introduction

Stem/progenitor cells are a type of undifferentiated cells or primitive cells that have the ability to replicate themselves and differentiate into multiple types of cells [1]. The VW-S/PC system plays an indispensable role in the development, maintenance, repair, and remodeling of blood vessels. It is reported that there are four major types of progenitor/stem cells in vascular tissues, including smooth muscle progenitor cells (SMPCs), endothelial progenitor cells (EPCs), myeloid progenitor cells, mesenchymal stem cells (MSCs), and pericytes [2–4]. As stem cells perform their functions, the microenvironment is extremely important in various physiologic and pathologic responses [2]. The microenvironment refers to the surrounding structures and components that can precisely regulate the dynamic balance of stem/progenitor cells [3], including nearby nerve cells, stromal cells, various growth factors, and cytokines bound to the extracellular matrix. Stem cell niche provides a dynamic microenvironment to maintain the tissue homeostasis and facilitate repair and regeneration.

Stem/progenitor cells are involved in the regulation and maintenance of vascular homeostasis under both physiological and pathophysiological conditions. The vascular wall provides a microenvironment to support and regulate VW-S/PCs. Multiple interactions between stem cell intrinsic factors, supporting cells, extracellular matrix, and signaling pathways specify cell fate and regulate stem cell proliferation and differentiation [5]. During vascular injury, stem/progenitor cells can be mobilized to the damaged area and differentiate into mature vascular wall cells, participating in the regulation of vascular development, repair, and remodeling [6]. Cardiovascular disease is the leading cause of death worldwide. The occurrence and development of cardiovascular diseases are closely related to the imbalance of vascular homeostasis and pathological vascular remodeling. Accumulating studies have demonstrated that the interaction between vascular microenvironment and VW-S/PCs is critical to vascular homeostasis.

Many studies have shown that some tissues around the blood vessel wall, such as nerve tissue, lymphatic tissue, adipose tissue, and vasoactive substances, are involved in the regulation of VW-S/PCs. Currently, how the microenvironmental factors regulate the function of VW-S/PCs remains to be clarified. Therefore, in this review, we highlight the key factors that regulate the functions of VW-S/PCs and discuss the interplay between VW-S/PCs and the microenvironmental homeostasis. Improved knowledge on the interactions will enhance the insight into VW-S/PCs behavior and the influence of the microenvironment on VW-S/PCs regenerative capability [4].

## 2. Tissues in the Microenvironment Affecting VW-S/PCs

There are many microenvironmental factors that affect VW-S/PCs, which together maintain the dynamic balance around the blood vessels. In this part, we will elaborate from the following main aspects, so as to understand the interaction among them (Figure 1).

### 2.1. Nerve Tissue

On the cross section of the blood vessel, nerve fibers are mainly distributed at the junction of the media and adventitia, and some nerves extend into the smooth muscle layer of the media. The reticular nerve plexus surrounding the blood vessel wall can be observed by specific staining. Normally, the density of nerve distribution on the artery wall is more abundant than that of vein [6]. It is reported that the activity of VW-S/PCs is affected by the nerve tissue surrounding the blood vessel wall [7–11]. It has been demonstrated that nerve growth factors (NGF) can promote EPC activation, mobilization, and endothelialization of tissue-engineered blood vessels [7]. In vitro, NGF promoted EPC proliferation and migration, form more colonies, and differentiate into endothelial cells (ECs). Flow cytometry analysis showed that the number of EPCs in peripheral circulation increased after NGF treatment in C57BL/6 mice [8]. The mobilization and homing of EPCs are essential for the development of antistenosis and antithrombosis tissue engineering blood vessels. When endothelial damage is severe, EPCs can migrate into the damaged site, where they differentiate into cells that substitute apoptotic ECs. The process can promote blood vessel reendothelialization and angiogenesis, lowering neointimal hyperplasia and thrombosis [9]. Stocum believed that nerves and the apical epidermal cap (AEC) together play a vital role in the proliferation of MSCs to form the blastema of regenerative amphibian limbs [10]. In addition, adult MSCs have shown increased nerve regeneration. Recent work also suggests that multipotent progenitor cells (MPCs) would possibly deliver neurotrophic advantages via indirect means, as MPCs exhibit the potential to manipulate their nearby proteolytic microenvironment [11].

### 2.2. Adipose Tissue

Adipose tissue is an organ with metabolism, regulation, and high regeneration potential. The adventitia of vascular wall is surrounded by a special kind of adipose tissue, called perivascular adipose tissue (PVAT) [12]. PVAT is a key regulator of vascular function, which plays a vital role in the expansion and differentiation of VW-S/PCs. Dysfunction of PVAT can promote vascular dilation and regulate further biological processes, including stem/progenitor cell activation, extracellular matrix remodeling, and angiogenesis [12]. Adult PVAT has the physiological characteristics of both white adipose tissue and brown adipose tissue. Its metabolic activity may affect vascular tension, vascular remodeling, angiogenesis, and thermogenesis [13]. VW-S/PCs in adipose tissue is the source of MSCs, commonly known as vascular wall resident MSCs or tissue-specific MSCs [14]. PVAT is considered as a supporting component of blood vessels and acts as a protective cushion on the walls of blood vessels from adjacent tissues during vessel relaxation and contraction [15]. It can be assumed that PVAT regulates vascular function and differentiation of VW-S/PCs by acting directly on vascular smooth muscle cells (VSMCs) and ECs through different mechanisms [16]. PVAT exists in the adventitia of most vessels and plays an essential role in maintaining vascular homeostasis. There is increasing evidence that PVAT, in response to intravascular mechanical injury, may release vasoactive substances that affect vascular function and regulate subsequent neointima formation by promoting VSMCs growth, adventitial inflammation, and neovascularization [17]. It can be speculated that the process involves the migration and differentiation of VW-S/PCs. Most studies ascribed that the role of PVAT in vascular remodeling is related to adipokines secreted by perivascular adipocytes. PVAT attached tightly to the walls of blood vessels and acted on them by paracrine adipokines, unlike other adipose tissues that required blood to transport adipokines [12–17]. However, Gu et al.'s research shows that MSCs also exist in PVAT and play a role in vascular regeneration. They immediately determined the heterogeneous PVAT-derived mesenchymal stem cells (PV-ADSCs) at a single-cell level and two subpopulations with distinct signaling pathways and signature genes by means of single-cell RNA-sequencing [18]. The characteristics of PVAT in angiogenesis are partly attributed to the fact that PVAT is an active tissue surrounding blood vessels and is regulated by the feedback of ECs and SMCs. Furthermore, numerous studies have shown that PVAT plays a protective role against atherosclerosis under physiological condition, by increasing the adiponectin level and eNOS expression, thereby inhibiting plaque formation, reducing inflammation, and improving endothelial function [19]. However, under pathophysiological conditions, these dysfunctional PVAT releases proinflammatory adipokines, resulting in the dysregulated calcium and phosphate homeostasis and enhanced vascular calcification and arterial stiffening [15, 20, 21]. Thus, the balance between pro- and anti-inflammatory adipokines secreted from adipocytes determines the effects of PVAT on vascular remodeling processes.

### 2.3. Lymphoid Tissue

Lymphoid tissue is also known as immune tissue, which plays a major role in the mucosal local anti-infective immunity [22]. In addition, lymphoid tissue and lymphocytes have some effect on the physiological and pathological activities of VW-S/PCs. Lymphocytes include B cells and T cells. In addition, there are other immune cells involved in the regulation of microenvironment, such as natural killer (NK) cells, macrophages, and dendritic cells [23]. Studies have proven that CD8^+^ T cells in favorable acute myeloid leukemia (AML) facilitated the growth of leukemia stem/progenitor cells (LSPCs) by way of stimulating the autocrine manufacturing of necessary hematopoietic cytokines such as interleukin-3 (IL-3). In contrast, LSPCs in aggressive AML are promoted by activating stem cells or proliferation-related pathways and promoting the expression of bone marrow (BM) CD8^+^ T cells [23]. Interactions between extracellular matrix elements, adhesion molecules, and cytokines may also provide the basis for fluid accumulation in vascular-associated lymphoid tissue areas and for practical improvement of subsequent atherosclerotic lesions [24]. This mechanism may also be involved in the activity of VW-S/PCs. Adaptive immunity is critical in vascular remodeling following arterial injury. P. Maga et al. hypothesized that acute changes in T cells at the site of percutaneous transluminal angioplasty (PTA) could be an indicator of their potential interaction with the injured vascular wall [25]. Thus, it used to be concluded that the observed acute reduction in T cells might be due to cell adhesion to the injured vascular wall. This change can affect the immune response to early vascular injury [26]. In addition, allogeneic T cells from corneal graft hosts may promote vascular ECs proliferation through vascular endothelial growth factor (VEGF) signaling pathway, while IFN-*γ* has shown an antiangiogenesis effect. T cells are important agents of angiogenesis in transplantation [27]. Besides, NK cells are known to be involved in vascular remodeling and intimal hyperplasia formation. The vascular remodeling in C57BL/6 NKC in CMV1(R) mice most likely be stimulated by activating IFN-*γ* secretion in NK cells [27]. Therefore, lymphatic tissue and lymphocytes may have an effect on VW-S/PCs. The underlying mechanism remains to be further studied.

## 3. Cytokines and Vasoactive Substances in the Microenvironment Affecting VW-S/PCs

There are cytokines and vasoactive substances that play equally important roles in the regulation of VW-S/PCs, including inflammatory factors, cytokines and peptides, extracellular matrix, thromboxane A2 (TXA2), histamine, 5-hydroxytryptamine (5-HT), and bradykinin (BK) (Figure 2). We will give an overview in this section.

### 3.1. Inflammatory Factors

Inflammatory factors, especially proinflammatory cytokines, play a direct or indirect role in the proliferation and differentiation of VW-S/PCs. It has been well known that tumor necrosis factor (TNF) is a proinflammatory cytokine that inhibits or promotes the migration and differentiation of VW-S/PCs. Elaboration of TNF is a very early event in development of ischemia/reperfusion injury [28]. It has been suggested that TNF-*α* significantly inhibited the proliferation, migration, adhesion, and vasculogenesis of late EPCs. TNF-*α* decreased the levels of NO secretion and KLF2 expression in EPCs at mRNA and protein levels but increased the levels of inflammatory factors along with ICAM-1 and MCP-1 [29]. Short-term treatment with anti-TNF used to be in a position to expand circulating EPCs while reducing disease process. This suggests that inhibiting the prevalence of inflammatory process may additionally positively have an effect on the endothelial feature [30]. However, Wang et al. suggested that overexpression of IL-10 had no impact on adhesion, migration, proliferation, tubule formation, and cell growth of EPCs. While after EPCs had been incubated with TNF-*α*, the overexpression of IL-10 could improve the EPCs function by activating the STAT3 signal pathway [31]. Likewise, it has additionally been confirmed that TNF-*α* regulates the apoptosis of human VSMCs and promoted the destabilization of atherosclerotic plaques with the aid of downregulating connexins 43 (Cx43) [32]. In addition, human bone marrow MSCs promote osteoblastic proliferation, migration, differentiation, and calcification in cytokine-activated inflammation [33]. In burn-induced heterotopic ossification, inflammatory factors including TNF-*α* can promote osteogenesis of adipose-derived MSCs in burn-injured mice [34]. The preceding research confirmed that fibrinogen and fibrin degradation merchandise produce a seasoned inflammatory impact on VSMCs through inducing the production of interleukin 6 (IL-6), TNF-*α*, and inducible nitric oxide synthase (iNOS) [35]. It has been shown that stromal cell-derived factor 1 (SDF-1) is able to regulate cell traffic and homing through chemokine receptor 4 (CXCR4), which plays an essential role in the recruitment of MSCs to target cells [36]. Altogether, these studies suggested that inflammatory factors could regulate the activity of VW-S/PCs.

### 3.2. Cytokines and Peptides

Many cytokines regulate the proliferation, migration, and differentiation of VW-S/PCs, including growth factors, chemokines, hormones, and some small molecules. Studies have shown that the migration of VW-S/PCs induced by SMC-derived chemokine (C-X-C motif) ligand 1 and chemokine (C-C motif) ligand 2 contributes to the formation of neointima, which act by means of CXCR2/Rac1/p38 and CCR2/Rac1/p38 signaling pathways [37]. In addition, sirolimus may stimulate the migration and differentiation of VW-S/PCs into SMCs through extracellular signal-regulated kinase (ERK)/epidermal growth factor receptor/*β*-catenin signaling pathway [38]. VEGF-A promotes the formation of new blood vessels by way of actively recruiting circulating EPCs [39]. VEGF-A plays a key role in human MSC-mediated myocardial regeneration. Homocysteine (Hcy) may affect epigenetic regulation of platelet-derived growth factor (PDGF) through demethylation of its promoter region through PDGF dependent signaling pathway, thereby stimulating proliferation of VSMCs [40]. This process may indirectly activate SMPCs on the vascular walls. Typical Wnt signaling performs a vital position in angiogenesis and regulation of EPCs viability. Mitochondrial biogenesis and function in EPCs could be mediated by Wnt signaling, which further reduced EPCs stemness and promoted EPCs differentiation. This process may contribute to pathologic vascular remodeling [41]. Platelet-derived microbubbles have been reported to promote EPCs proliferation by delivering TGF-*β*1 [42]. Nana et al. found that HDL ApoAI analog peptide reverse D-4F (Rev-D4F) might amplify the volume of EPCs by increasing SDF-1*α* level and decreasing TNF-*α* level in peripheral blood of C57BL/6J mice induced by high-fat diet. In addition, EPCs dysfunction induced by TNF-*α* was partially restored by stimulating phosphatidylinositol 3 kinase (PI3K)/AKT signaling pathway [43]. In addition, previous studies have reported that estrogen inhibits VSMCs osteogenic differentiation in vitro and arterial calcification in vivo by promoting autophagy [44], while in postmenopausal women with osteoporosis treated with estrogen, the mRNA expression of estrogen receptor and alkaline phosphatase (ALP) increased, suggesting that estrogen may have a significant effect on osteoblastic differentiation of bone marrow MSCs in women with osteoporosis [45]. The C3H/10T1/2 mesenchymal stem cell line itself secretes cytokines, such as insulin-like growth factor-1 (IGF-1), which help regulate tissue regeneration [46]. Therefore, multiple cytokines are associated with enhanced function in both circulating stem/progenitor cells and VW-S/PCs.

### 3.3. Extracellular Matrix

The extracellular matrix (ECM) is an intricate network of macromolecules with distinctive physical, biochemical, and biomechanical properties, providing essential physical scaffolding for the cellular morphogenesis, migration, differentiation, and homeostasis [47, 48]. The main components of ECM consist of collagen, glycoprotein, elastic protein, amino glucan, and proteoglycans. ECM may play an important role in maintaining the normal function of VW-S/PCs. Costa et al. reported that ECM, nearby microenvironment parameters, and cell-cytokine interactions are involved in controlling quiescence, self-renewal, and differentiation of hematopoietic stem/progenitor cells (HSPCs) [49]. In addition, the ECM-coated stents enabled endothelial regeneration and inhibited neointimal growth, which indicated that ECM coating effectively promoted the adhesion and proliferation of EPCs and had selectively opposite effects on SMCs [50]. Allen et al. have shown that human EPCs and MSCs can form microvascular networks in fibrin, type I collagen, and engineered peptide hydrogel PuraMatrix within seven days in immunodeficient mice. The results showed that ECM provides a suitable environment for human EPCs and MSCs to form new vascular networks [51]. VSMCs are uncovered to a range of mechanical signals, inclusive stiffness, and stretching of vascular ECM, which are concerned in the rules of VSMC contraction. ECM softening performs a key position in the transformation of VSMCs from contractile to proliferative and gives a conceivable goal for the therapy of VSMCs dysfunction and aortic dissection disease [52]. Although few studies have studied the direct regulation of ECM on VW-S/PCs, the effect can be indirectly deduced by other cellular mechanisms.

### 3.4. Vasoactive Substances

Vasoactive substances, including vasoconstrictors and vasodilators, are a group of secreted mediators and other signaling molecules released by the tissues [53]. The more obvious effect of these factors is that they can act directly on vascular smooth muscle along with blood circulation, including thromboxane A2 (TXA2), histamine, 5-hydroxytryptamine (5-HT), and bradykinin (BK) [54]. It has been suggested that *in vitro*, histamine did not stimulate proliferation of cultured SMCs by itself but enhanced PDGF-induced cell proliferation through a mechanism impartial of H1 and H2 histamine receptors [55]. Moreover, Liu et al. verified that activation of 5-HT2BR and *β*-arrestin2-based downstream signaling was key pathological processes in neointimal formation, and 5-HT2BR may additionally be an attainable goal for the therapeutic intervention of vascular restenosis [56]. It has been well demonstrated that resident VW-S/PCs could differentiate into ECs and SMCs, contributing to intimal accumulation during the process of vascular remodeling, such as neointimal hyperplasia and atherosclerosis. Therefore, the vasoactive substances might play an important role in the mobilization, migration, and differentiation of VW-S/PCs, thereby to regulate the vascular function.

## 4. Biochemical Signals in the Microenvironment Affecting VW-S/PCs

VW-S/PCs play an important role in the pathological development of various cardiovascular diseases through migration and differentiation. After being stimulated by vascular injury, VW-S/PCs migrate to the intima and differentiate into vascular cells to participate in the formation of neointima. It was reported that VW-S/PCs once activated were mobilized to the site of injury or other lesions. During this process, a variety of chemokines, chemokine structural analogues, and downstream signals related to the activation of paracrine cytokines contribute to the development or regeneration of VW-S/PCs [57]. Studies have revealed successively that many biochemical cues, such as ERK and PI3K/AKT signaling, Rac1/Cdc42 signaling pathway, and Wnt and Notch signaling pathway, are involved in the regulation of stem cell migration and differentiation under physiological and pathological condition [57–60]. For example, Dickkopf-3 (DKK3), a secreted glycoprotein, can activate ERK1/2, PI3K/AKT, Rac1, and RhoA signaling pathways by binding to chemokine (C-X-C motif) ligand 7 (CXCR7), to regulate the migration of Sca-1^+^ vascular stem cells in the vascular adventitia. Tissue-engineered vascular grafts loaded with DKK3 can effectively endothelialize and recruit progenitor cells, thereby affecting vascular remodeling [58]. Furthermore, the elevated leptin in the vascular wall and circulation after vascular injury could activate leptin receptor-dependent STAT3-Rac1/Cdc42-ERK-FAK signaling to enhance the migration of Sca-1^+^ progenitor cells and the formation of neointima [59]. Recently, it was suggested that MSCs could promote EPCs migration and vascularization in tissue engineering structures by activating CXCR2-Src-PKL/Vav2-Rac1 pathways [61]. In addition, macrophage-derived matrix metalloproteinase 8 (MMP8) could promote the differentiation of VW-S/PCs into SMCs through modulating the activity of transforming growth factor-*β* (TGF-*β*) and metalloproteinase domain protein 10- (ADAM10-) Notch1 signaling pathway to contribute to vascular injury induced neointimal hyperplasia [57]. Collectively, the migration or differentiation of VW-S/PCs is a complicated process, which is closely related to the regulation of biochemical signals. Therefore, understanding the regulatory mechanism involved in the migration and differentiation of VW-S/PCs under pathological conditions is fundamental for exploring the occurrence and development of related cardiovascular diseases.

## 5. Organoid and Stem Cell Niche

Organoids are stem cell-derived 3D cell culture systems which accurately mimic *in vivo* mature organ architecture and associated tissue microenvironments. Organoids facilitate the systematic experimental manipulation to identify and characterize stem cell niche interactions and uncover new niche components [62]. As an emerging research model *in vitro*, organoids have achieved major progress in recapitulating morphological aspects of organs and personalized precision therapy [63]. For many tissues, single resident stem cells growing *in vitro* under appropriate 3D conditions can produce products called organoids. These tissues summarize much of the cellular composition and structure of the organs in the body from which they derive, including the formation of stem cell niches [62]. These organoids can be derived from embryonic stem cells (ESCs), induced pluripotent stem cells (iPSCs), or tissue resident adult stem cells. In many cases, the stem cell niche, rather than the stem cell itself, controls the fate of the cell. For example, Booth et al. have shown that transplanting single neural stem cells into the mammary gland microenvironment can reprogram them into mammary epithelial cells of regenerative mammary epithelial trees [64]. The use of organoid culture can help identify important niche components and gain a deeper understanding of how stem cell niche controls cell activity. Sato et al. experimentally identified Paneth cells as key members of the intestinal stem cell niche [65], which contain an abundance of antimicrobial peptides and immunomodulating proteins to mediate intestinal stem cell renewal and regeneration following homeostasis or injury. Such experiments in other tissues will help identify cell types that constitute the smallest ecological niche, the components necessary for stem cell maintenance and tissue self-renewal. Additionally, coculturing of pluripotent stem cells, MSCs, and ECs on 3D matrix is developing rapidly, forming a new model for the evolution of vascularized organoids with blood perfusion [63]. Therefore, the vascularization organoids are conducive to composing a functional communication niche and exhibit the physiological function comprehensively.

## 6. Conclusions and Perspectives

VW-S/PCs are a vital source of all sorts of vascular cells needed to maintain, build, repair, and remodel blood vessels. VW-S/PCs, therefore, play quintessential roles in the development, normal physiology, and pathophysiology of numerous diseases. There are many kinds of microenvironmental factors that affect the function of VW-S/PCs. Microenvironmental factors might do not act on the vessels solely or directly, but a variety of factors cooperate to regulate the VW-S/PCs. The biochemical effects of many microenvironmental factors are dependent on background conditions, and these factors may intersect to form a minimal structural and functional unit that modulates homeostasis of VW-S/PCs physiological function. Currently, the role of microenvironmental factors in the activation, mobilization, migration, and differentiation of VW-S/PCs is largely unknown. More research is needed to obtain a higher appreciation of the physiological and pathological functions and potential mechanisms of the surrounding microenvironment of VW-S/PCs, which will help reveal the full therapeutic potential of VW-S/PCs in treating human diseases.

## Figures and Tables

**Figure 1:** Proposed model of microenvironment in vascular stem cells niche. The vessel wall comprises an inner layer (intima), a thicker media layer (smooth muscle cells), and an outer layer (adventitia). The intima is mainly composed of a monolayer of endothelial cells (ECs), including mature and terminally differentiated cells (pink) and also endothelial progenitor cells (EPCs) (blue), which can proliferate, migrate, and differentiate into ECs to replace injured ECs in vascular repair. The adventitia is a dynamic layer in active communication with the other vessel wall layers, and it contains various cell types among others, including PCs (CD34^+^/SCa-1^+^ progenitor cells), mesenchymal stem cells (MSCs), macrophages, fibroblasts, adipocytes, pericytes, lymphocytes (B cells and T cells), and NK cells surrounding the neural fibers, lymphatic vessels, and secreted signaling molecules in adventitia.

**Figure 2:** Multiple signaling pathways are involved in the migration of VW-S/PCs. Under physiological conditions, VW-S/PCs reside in the microenvironment “stem cell niche.” In vascular diseases, inflammatory factors, cytokines, and chemokines are released by activated VW-S/PCs. IL-10 affects intracellular expression of related genes through JAK-STAT pathway, and SOCS is a specific inhibitor of the pathway. Vascular Sca-1^+^ cell migration can be induced by SMC-derived chemokine CCR2 and CXCR2 through the CCR2/Rac1/P38 and CXCR2/Rac1/P38 signaling pathways. Extracellular matrix (ECM) induces phenotypic transformation and cytoskeletal changes and affects the intracellular pH balance, providing a potential target for vascular diseases.

## References

[1] Mauretti A., Spaans S., Bax N. A. M., Sahlgren C., Bouten C. V. C. (2017). Cardiac progenitor cells and the interplay with their microenvironment. *Stem Cells International*.

[2] Zhang L., Issa Bhaloo S., Chen T., Zhou B., Xu Q. (2018). Role of resident stem cells in vessel formation and arteriosclerosis. *Circulation Research*.

[3] Clara J. A., Monge C., Yang Y., Takebe N. (2020). Targeting signalling pathways and the immune microenvironment of cancer stem cells - a clinical update. *Nature Reviews. Clinical Oncology*.

[4] Oya Y., Hayakawa Y., Koike K. (2020). Tumor microenvironment in gastric cancers. *Cancer Science*.

[5] Mannino G., Russo C., Maugeri G. (2022). Adult stem cell niches for tissue homeostasis. *Journal of Cellular Physiology*.

[6] Saeed P., Tavakoli Rad S., Bisschop P. (2018). Dysthyroid optic neuropathy. *Ophthalmic Plastic & Reconstructive Surgery*.

[7] Zeng W., Yuan W., Li L. (2010). The promotion of endothelial progenitor cells recruitment by nerve growth factors in tissue-engineered blood vessels. *Biomaterials*.

[8] Fang J., Huang X., Han X. (2020). Endothelial progenitor cells promote viability and nerve regenerative ability of mesenchymal stem cells through PDGF-BB/PDGFR-beta signaling. *Aging (Albany NY)*.

[9] Fang J. F., Huang X. N., Han X. Y. (2018). Combined transplantation of mesenchymal stem cells and endothelial progenitor cells restores cavernous nerve injury-related erectile dysfunction. *The Journal of Sexual Medicine*.

[10] Stocum D. L. (2019). Nerves and proliferation of progenitor cells in limb regeneration. *Developmental Neurobiology*.

[11] Lozito T. P., Jackson W. M., Nesti L. J., Tuan R. S. (2014). Human mesenchymal stem cells generate a distinct pericellular zone of MMP activities via binding of MMPs and secretion of high levels of TIMPs. *Matrix Biology*.

[12] Tinajero M. G., Gotlieb A. I. (2020). Recent developments in vascular adventitial pathobiology: the dynamic adventitia as a complex regulator of vascular disease. *The American Journal of Pathology*.

[13] Mancio J., Oikonomou E. K., Antoniades C. (2018). Perivascular adipose tissue and coronary atherosclerosis. *Heart*.

[14] Meyers C. A., Xu J., Asatrian G. (2018). WISP-1 drives bone formation at the expense of fat formation in human perivascular stem cells. *Scientific Reports*.

[15] Hu H., Garcia-Barrio M., Jiang Z. S., Chen Y. E., Chang L. (2021). Roles of perivascular adipose tissue in hypertension and atherosclerosis. *Antioxidants & Redox Signaling*.

[16] Zhang Y. Y., Shi Y. N., Zhu N. (2021). PVAT targets VSMCs to regulate vascular remodelling: angel or demon. *Journal of Drug Targeting*.

[17] Horimatsu T., Kim H. W., Weintraub N. L. (2017). The role of perivascular adipose tissue in non-atherosclerotic vascular disease. *Frontiers in Physiology*.

[18] Gu W., Nowak W. N., Xie Y. (2019). Single-cell RNA-sequencing and metabolomics analyses reveal the contribution of perivascular adipose tissue stem cells to vascular remodeling. *Arteriosclerosis, Thrombosis, and Vascular Biology*.

[19] Carbone F., Mach F., Montecucco F. (2015). The role of adipocytokines in atherogenesis and atheroprogression. *Current Drug Targets*.

[20] Qi X. Y., Qu S. L., Xiong W. H., Rom O., Chang L., Jiang Z. S. (2018). Perivascular adipose tissue (PVAT) in atherosclerosis: a double-edged sword. *Cardiovascular Diabetology*.

[21] Shields K. J., Barinas-Mitchell E., Gingo M. R. (2013). Perivascular adipose tissue of the descending thoracic aorta is associated with systemic lupus erythematosus and vascular calcification in women. *Atherosclerosis*.

[22] Jaeger-Ruckstuhl C. A., Hinterbrandner M., Hopner S. (2020). TNIK signaling imprints CD8(+) T cell memory formation early after priming. *Nature Communications*.

[23] Radpour R., Riether C., Simillion C., Hopner S., Bruggmann R., Ochsenbein A. F. (2019). CD8^+^ T cells expand stem and progenitor cells in favorable but not adverse risk acute myeloid leukemia. *Leukemia*.

[24] Millonig G., Schwentner C., Mueller P., Mayerl C., Wick G. (2001). The vascular-associated lymphoid tissue: a new site of local immunity. *Current Opinion in Lipidology*.

[25] Maga P., Mikolajczyk T. P., Partyka L. (2018). Involvement of CD8+ T cell subsets in early response to vascular injury in patients with peripheral artery disease in vivo. *Clinical Immunology*.

[26] Di Zazzo A., Tahvildari M., Subbarayal B. (2017). Proangiogenic function of T cells in corneal transplantation. *Transplantation*.

[27] de Vries M. R., Seghers L., van Bergen J. (2013). C57BL/6 NK cell gene complex is crucially involved in vascular remodeling. *Journal of Molecular and Cellular Cardiology*.

[28] Solovey A., Somani A., Belcher J. D. (2017). A monocyte-TNF-endothelial activation axis in sickle transgenic mice: therapeutic benefit from TNF blockade. *American Journal of Hematology*.

[29] Chu H., Li H., Guan X. (2018). Resveratrol protects late endothelial progenitor cells from TNF-alpha-induced inflammatory damage by upregulating Kruppel-like factor-2. *Molecular Medicine Reports*.

[30] Spinelli F. R., Metere A., Barbati C. (2013). Effect of therapeutic inhibition of TNF on circulating endothelial progenitor cells in patients with rheumatoid arthritis. *Mediators of Inflammation*.

[31] Wang Y., Chen Q., Zhang Z., Jiang F., Meng X., Yan H. (2015). Interleukin-10 overexpression improves the function of endothelial progenitor cells stimulated with TNF-*α* through the activation of the STAT3 signaling pathway. *International Journal of Molecular Medicine*.

[32] Tang M., Fang J. (2017). TNF-*α* regulates apoptosis of human vascular smooth muscle cells through gap junctions. *Molecular Medicine Reports*.

[33] Chen Q., Shou P., Zheng C. (2016). Fate decision of mesenchymal stem cells: adipocytes or osteoblasts?. *Cell Death & Differentiation*.

[34] Li C., Li G., Liu M., Zhou T., Zhou H. (2016). Paracrine effect of inflammatory cytokine-activated bone marrow mesenchymal stem cells and its role in osteoblast function. *Journal of Bioscience and Bioengineering*.

[35] Lu P., Liu J., Pang X. (2015). Pravastatin inhibits fibrinogen- and FDP-induced inflammatory response via reducing the production of IL-6, TNF-*α* and iNOS in vascular smooth muscle cells. *Molecular Medicine Reports*.

[36] Chen L., Zou X., Zhang R. X. (2016). IGF1 potentiates BMP9-induced osteogenic differentiation in mesenchymal stem cells through the enhancement of BMP/Smad signaling. *BMB Reports*.

[37] Yu B., Wong M. M., Potter C. M. (2016). Vascular stem/progenitor cell migration induced by smooth muscle cell-derived chemokine (C-C Motif) ligand 2 and chemokine (C-X-C motif) ligand 1 contributes to neointima formation. *Stem Cells*.

[38] Wong M. M., Winkler B., Karamariti E. (2013). Sirolimus stimulates vascular stem/progenitor cell migration and differentiation into smooth muscle cells via epidermal growth factor receptor/extracellular signal-regulated kinase/*β*-catenin signaling pathway. *Arteriosclerosis, Thrombosis, and Vascular Biology*.

[39] Yang L., Du J., Hou J., Jiang H., Zou J. (2011). Platelet factor-4 and its p 17-70 peptide inhibit myeloma proliferation and angiogenesis in vivo. *BMC Cancer*.

[40] Han X. B., Zhang H. P., Cao C. J. (2014). Aberrant DNA methylation of the PDGF gene in homocysteine-mediated VSMC proliferation and its underlying mechanism. *Molecular Medicine Reports*.

[41] Shao Y., Chen J., Freeman W. (2019). Canonical Wnt signaling promotes neovascularization through determination of endothelial progenitor cell fate via metabolic profile regulation. *Stem Cells*.

[42] Yan J., Bao H., Fan Y. J., Jiang Z. L., Qi Y. X., Han Y. (2020). Platelet-derived microvesicles promote endothelial progenitor cell proliferation in intimal injury by delivering TGF‐*β*1. *The FEBS Journal*.

[43] Nana Y., Peng J., Jianlin Z. (2015). Reverse-D-4F increases the number of endothelial progenitor cells and improves endothelial progenitor cell dysfunctions in high fat diet mice. *PLoS One*.

[44] Peng Y. Q., Xiong D., Lin X. (2017). Oestrogen inhibits arterial calcification by promoting autophagy. *Scientific Reports*.

[45] Kim H. Y., Lee Y., Yoon H. S. (2021). A novel method to differentiate tonsil-derived mesenchymal stem cells in vitro into estrogen-secreting cells. *Tissue Engineering and Regenerative Medicine*.

[46] Witt R., Weigand A., Boos A. M. (2017). Mesenchymal stem cells and myoblast differentiation under HGF and IGF-1 stimulation for 3D skeletal muscle tissue engineering. *BMC Cell Biology*.

[47] Kai F., Drain A. P., Weaver V. M. (2019). The extracellular matrix modulates the metastatic journey. *Developmental Cell*.

[48] Marchand M., Monnot C., Muller L., Germain S. (2019). Extracellular matrix scaffolding in angiogenesis and capillary homeostasis. *Seminars in Cell & Developmental Biology*.

[49] Costa M. H. G., de Soure A. M., Cabral J. M. S., Ferreira F. C., da Silva C. L. (2018). Hematopoietic niche-exploring biomimetic cues to improve the functionality of hematopoietic stem/progenitor cells. *Biotechnology Journal*.

[50] Kokeny G., Calvier L., Legchenko E., Chouvarine P., Mozes M. M., Hansmann G. (2020). PPAR*γ* is a gatekeeper for extracellular matrix and vascular cell homeostasis. *Current Opinion in Nephrology and Hypertension*.

[51] Allen P., Melero-Martin J., Bischoff J. (2011). Type I collagen, fibrin and PuraMatrix matrices provide permissive environments for human endothelial and mesenchymal progenitor cells to form neovascular networks. *Journal of Tissue Engineering and Regenerative Medicine*.

[52] Shao Y., Li G., Huang S. (2020). Effects of extracellular matrix softening on vascular smooth muscle cell dysfunction. *Cardiovascular Toxicology*.

[53] Jaimes L., Vinet R., Knox M. (2019). A review of the actions of endogenous and exogenous vasoactive substances during the estrous cycle and pregnancy in rats. *Animals*.

[54] Machida T., Iizuka K., Hirafuji M. (2013). 5-hydroxytryptamine and its receptors in systemic vascular walls. *Biological & Pharmaceutical Bulletin*.

[55] Kimura S., Noguchi H., Nanbu U., Wang K. Y., Sasaguri Y., Nakayama T. (2018). Relationship between CCL22 expression by vascular smooth muscle cells and macrophage histamine receptors in atherosclerosis. *Journal of Atherosclerosis and Thrombosis*.

[56] Liu Y., Wang Z., Li J. (2018). Inhibition of 5-hydroxytryptamine receptor 2B reduced vascular restenosis and mitigated the beta-arrestin2-mammalian target of rapamycin/p70S6K pathway. *Journal of the American Heart Association*.

[57] Yang F., Chen Q., Yang M. (2020). Macrophage-derived MMP-8 determines smooth muscle cell differentiation from adventitia stem/progenitor cells and promotes neointima hyperplasia. *Cardiovascular Research*.

[58] Issa Bhaloo S., Wu Y., Le Bras A. (2018). Binding of Dickkopf-3 to CXCR7 enhances vascular progenitor cell migration and degradable graft regeneration. *Circulation Research*.

[59] Zhang T., Yang P., Li T., Gao J., Zhang Y. (2019). Leptin expression in human epicardial adipose tissue is associated with local coronary atherosclerosis. *Medical Science Monitor: International Medical Journal of Experimental and Clinical Research*.

[60] Li L., Ren S., Hao X., Zhen Z., Ji L., Ji H. (2021). MicroRNA-29b inhibits human vascular smooth muscle cell proliferation via targeting the TGF-beta/Smad3 signaling pathway. *Experimental and Therapeutic Medicine*.

[61] Li Z., Yang A., Yin X. (2018). Mesenchymal stem cells promote endothelial progenitor cell migration, vascularization, and bone repair in tissue-engineered constructs via activating CXCR2-Src-PKL/Vav2-Rac1. *The FASEB Journal*.

[62] Murrow L. M., Weber R. J., Gartner Z. J. (2017). Dissecting the stem cell niche with organoid models: an engineering-based approach. *Development*.

[63] Yu J. (2021). Vascularized organoids: a more complete model. *International Journal of Stem Cells*.

[64] Booth B. W., Mack D. L., Androutsellis-Theotokis A., McKay R. D., Boulanger C. A., Smith G. H. (2008). The mammary microenvironment alters the differentiation repertoire of neural stem cells. *Proceedings of the National Academy of Sciences*.

[65] Sato T., van Es J. H., Snippert H. J. (2011). Paneth cells constitute the niche for Lgr5 stem cells in intestinal crypts. *Nature*.

